The article "Correlation between cigarette smoking and alcohol consumption and Rosacea: A two‐sample Mendelian randomization study" was retracted in 2025. Reasons: compromised peer review; unreliable results or conclusions; concerns about the methods.

# Correlation between cigarette smoking and alcohol consumption and Rosacea: A two‐sample Mendelian randomization study

**DOI:** 10.1111/srt.13765

**Published:** 2024-06-16

**Authors:** Juan Wang, Lingli Zhang

**Affiliations:** ^1^ Department of Otorhinolaryngology Central Hospital Affiliated to Chongqing University of Technology Chongqing China

**Keywords:** alcohol consumption, cigarette smoking, Mendelian randomization, risk, Rosacea

## Abstract

**Background:**

Controversy persists regarding the causal relationship between Cigarette smoking, alcohol consumption, and Rosacea. This paper employs the Mendelian randomization (MR) method to elucidate the correlation between Cigarette smoking, alcohol consumption, and Rosacea. The aim is to contribute valuable insights to aid in the prevention and early treatment of Rosacea.

**Method:**

Summary datasets for cigarette smoking parameters (Cigarettes smoked per day, Smoking status: Previous, smoking status: Current) and alcohol consumption (Alcoholic drinks per week) were selected alongside data for Rosacea from genome‐wide association studies (GWAS). The Two‐sample MR method was employed to analyze the correlation between cigarette smoking, alcohol consumption, and Rosacea. Various MR analysis methods, including inverse variance weighting (IVW), MR‐Egger, Simple Mode, Weighted Mode, and Weighted Median, were chosen. IVW served as the primary analysis method.

**Results:**

The results indicate a significant negative association between Cigarettes smoked per day and Rosacea. Moreover, a significant positive correlation was observed between Smoking status: Previous and Rosacea. However, no significant associations were found between Smoking status: Current, Alcoholic drinks per week, and Rosacea.

**Conclusion:**

This study provides further clarity on the association between cigarette smoking, drinking, and Rosacea through a two‐sample MR analysis. Notably, the number of cigarettes smoked per day appears to be associated with a reduced incidence of Rosacea, while cigarette smoking cessation may increase the risk. Surprisingly, alcohol consumption does not emerge as a significant risk factor for Rosacea. These findings contribute to a nuanced understanding of the complex relationship between lifestyle factors and the occurrence of Rosacea, offering potential insights for preventive measures and early intervention.

## 1 INTRODUCTION

Rosacea, a chronic inflammatory disease, impacts approximately 5% of the adult population.^1^ Its primary clinical manifestations include nasal flushing, inflammatory papules, and facial pustules.^2^ The related symptoms of rosacea seriously affect the psychological state of patients.^3^ Despite its prevalence, the precise mechanisms underlying Rosacea remain uncertain, with potential links to immune and neurovascular disorders,^4^ it may also be related to solar damage^5^ and demodex mites.^6^ Environmental triggers are also believed to contribute to Rosacea's development and progression.^7^ While previous studies have suggested potential associations between cigarette smoking, alcohol consumption, and Rosacea, the presence of various confounding factors has obscured the establishment of clear causal relationships.^8^, ^9^, ^10^

Cigarette smoking and alcohol consumption, recognized risk factors for diseases, significantly contribute to premature mortality.^11^ Cigarette smoking exerts an impact on various inflammatory diseases, including chronic obstructive pulmonary disease,^12^ periodontal disease,^13^ and psoriasis.^14^ Similarly, studies have identified associations between alcohol consumption and certain skin conditions.^15^ Conflicting findings have been reported regarding the impact of cigarette smoking on Rosacea, with some suggesting a potential reduction in prevalence,^16^ while others propose cigarette smoking and obesity as external triggers for Rosacea.^17^ The relationship between alcohol consumption and Rosacea is also debated, with some studies suggesting an association,^8^, ^18^ while others find no significant difference.^19^ Studies have shown that cigarette smoking and drinking can affect the human microbiome,^20^, ^21^ and changes in skin microbiome and intestinal microbiome are closely related to the occurrence and development of Rosacea.^22^, ^23^, ^24^ Effective treatment interventions targeting disturbed skin and gut microbiota in Rosacea patients have been documented.^25^ However, the unclear pathophysiological mechanisms of Rosacea underscore the importance of understanding its risk factors for preventive strategies and further exploration of its underlying mechanisms.

The article "Correlation between cigarette smoking and alcohol consumption and Rosacea: A two‐sample Mendelian randomization study" was retracted in 2025. Reasons: compromised peer review; unreliable results or conclusions; concerns about the methods.

To address these uncertainties, this study aims to investigate the associations between cigarette smoking (Cigarettes smoked per day, Smoking status: Previous, Smoking status: Current) and drinking (Alcoholic drinks per week) with Rosacea independently, utilizing Mendelian randomization (MR). MR offers a method to assess genetically predicted associations between exposure (smoking and alcohol consumption) and outcome (Rosacea), utilizing genetic variants as instrumental variables (IV). This approach involves correlating exposure single‐nucleotide polymorphisms (SNPs) from independent genome‐wide association studies (GWAS) data with outcome SNPs, aiming to clarify the causal relationship between the two traits.^26^ MR mitigates the limitations of traditional observational studies and minimizes the impact of confounding factors, thereby enhancing the credibility of the findings.

## 2 METHODS

### 2.1 Research design

In this study, we conducted multiple two‐sample MR Analyses using GWAS data from public databases to examine the associations of cigarette smoking and alcohol consumption with Rosacea. Three principles were followed in the MR analysis:^1^ the instrumental variables were strongly associated with exposure (*P* < 5 × 10^−8^ and *F* > 10^27^).^2^ the instrumental variables were associated with outcomes only by exposure;^3^ The instrumental variables should be independent of other confounding factors. Our MR analysis was conducted based on the three instrumental variable assumptions described above.^26^

### 2.2 Data source

The data used in this study were all obtained from publicly available GWAS with ethical approval and informed consent. We choose GWAS data from European descent from IEU GWAS database (https://gwas.mrcieu.ac.uk/) to download to cigarette smoking and drinking of data set and data set of Rosacea. The IEU database has acquired the Rosacea dataset from the Finngen database R5 version, comprising a total of 1195 cases and 211 139 controls. Additionally, GWAS datasets for “Cigarettes Smoked per Day” and “Alcoholic Drinks per Week” were sourced from the GWAS & Sequencing Consortium of Alcohol and Nicotine Use Genetic data collection, involving 249 752 and 335 394 participants respectively.^28^ The GWAS dataset related to smoking status was obtained from the Neale lab analysis of UK Biobank phenotypes, round 1 (Previous: n‐case = 118 419, n‐control = 217 605, Current: n‐case = 33 928, n‐control = 302 096) (data set details are provided in Table 1).

**TABLE 1:** The GWAS data source details in our study.

Phenotype	Data source	PMID	Case	Control	Sample size	Ancestry
Rosacea	Finngen		1195	211 139	212 334	European
Cigarettes smoked per day	GSCAN	30643251			249 752	European
Alcoholic drinks per week	GSCAN	30643251			335 394	European
Smoking status: Current	Neale Lab		33 928	302 096	336 024	European
Smoking status: Previous	Neale Lab		118 419	217 605	336 024	European

Abbreviation: GSCAN, GWAS and Sequencing Consortium of Alcohol and Nicotine use.

The diagnosis of Rosacea is established based on meeting the diagnostic criteria outlined by code L71 in the Tenth Revision of the International Statistical Classification of Diseases and Related Health Problems. To assess the quantity of cigarettes smoked per day, we employed a five‐point scale (≤5, 6–15, 16–25, 26–35, > 35) by asking subjects, “How many cigarettes do/did you smoke per day?” Similarly, to ascertain the average weekly alcohol consumption, we queried subjects, “Thinking about the past year, on average, how many drinks did you have each week?”. Cigarette smoking status (current or previous) was determined based on subjects' acknowledgment of having been exposed to at least 100 cigarettes in their lifetime.^29^

The article "Correlation between cigarette smoking and alcohol consumption and Rosacea: A two‐sample Mendelian randomization study" was retracted in 2025. Reasons: compromised peer review; unreliable results or conclusions; concerns about the methods.

### 2.3 Selection of genetic instruments

Using the Two SampleMR package in R^30^, the genome‐wide significance (*P* < 5 × 10^−8^) and without linkage disequilibrium (LD) (*r* ^2^ < 0.001 and 10 000 KB) were screened out and IVs with F<10 were deleted. If the associated SNPs were not available in the GWAS data, we simply removed the SNPs. Then we try to infer the positive chain alleles, using the allelic frequencies of the palindromes. We scrutinized these SNPs using PhenoScanner to address the phenotypes associated with each SNP and to minimize confounders,^31^ such as Inflammatory bowel diseas,^32^ serum 25‐hydroxyvitamin D.^33^ The SNPs associated with confounders and Rosacea outcomes were then manually screened and removed. Finally, we obtained the relevant SNPs for analysis (Supplementary Material 2 for detailed codes).

### 2.4 Statistical analysis

We combined MR estimates by using inverse variance weighting (IVW) as the primary method. MR‐Egger,^34^ Simple mode, Weighted mode, and weighted median methods^35^ were used as sensitivity analyses. IVW obtained a total estimate of the effect of exposure on the outcome by combining the causal estimate of Wald for each IV, and IVW was used as the primary analysis.^36^ The nonzero intercept values shown by the MR‒Egger method were mainly used to check for horizontal pleiotropy.^34^ The weighted median gives an accurate estimate based on the assumption that at least 50% of IVs are effective.^35^ The simple mode, weighted mode, and weighted median methods were mainly used to verify the reliability and stability of the results. we assessed causality using the odds ratio (OR) and 95% confidence interval (95% CI) to determine significance. To correct for the resulting *P*‐values, we applied a Benjamini‐Hochberg false discovery rates (FDR) correction.

Next, we executed the MR‐Egger method to obtain intercept values to evaluate horizontal pleiotropy. The Q statistic from Cochran's IVW was then utilized to investigate the impact of heterogeneity.

## 3 RESULT

After screening, a total of 22 SNPs were included in the analysis when Cigarettes smoked per day was used as exposure. When Smoking status: Current was used as exposure, a total of 15 SNPs were included in the analysis. When Smoking status: Previous was used as exposure, a total of 19 SNPs were included in the analysis. In the MR analysis of Alcoholic drinks per week and Rosacea, rs1260326, rs153106 were associated with Inflammatory bowel disease, so they were removed by us. A total of 31 SNPs were included in the analysis when Alcoholic drinks per week was used as exposure. All MR‐Egger analyses showed no horizontal pleiotropy (*P* > 0.05). All SNPs included in the analysis had F‐statistics greater than 10, indicating that they were all strong instrumental variables. In addition, no heterogeneity was found for all MR results (*P* > 0.05).

The article "Correlation between cigarette smoking and alcohol consumption and Rosacea: A two‐sample Mendelian randomization study" was retracted in 2025. Reasons: compromised peer review; unreliable results or conclusions; concerns about the methods.

The number of SNPs analyzed for all MR together with the associated MR results is presented in detail in Table 2. The results suggested that there was a significant negative association between Cigarettes smoked per day and Rosacea (IVW: OR = 0.664, 95% CI: 0.481– 0.918, *P* =** 0.013**, *P*‐value(After FDR correction) = **0.026**) results suggested a difference. There was a significant positive correlation between Smoking status: Previous and Rosacea(IVW: OR = 84.398, 95% CI: 4.040–1.76E+3, *P* = **0.004**, *P*‐value(After FDR correction) = **0.016**). No significant associations were found between Smoking status: Current (IVW: OR = 0.093, 95% CI: 4.26E‐4–20.498, *P* = 0.388, *P*‐value(After FDR correction) = 0.472) and Alcoholic drinks per week(IVW: OR = 1.489, 95% CI: 0.503–4.400, *P* = 0.472, *P*‐value (After FDR correction) = 0.472) and Rosacea (Figure 1).

**TABLE 2:** Results of MR analysis of smoking and drinking with Rosacea.

Exposure	Outcome	SNP	Method	OR	95% CI	*P*‐value	*P*‐value (After FDR correction)	Q_pval	*P*‐value (pleiotropy)
Cigarettes smoked per day	Rosacea	22	MR Egger	0.644	0.360–1.150	0.152		20(0.299)	
			Weighted median	0.809	0.522–1.253	0.343			
			Inverse variance weighted	0.664	0.481–0.918	**0.013**	**0.026**	21(0.354)	0.898
			Simple mode	0.904	0.341–2.392	0.841			
			Weighted mode	0.743	0.495–1.116	0.167			
Alcoholic drinks per week	Rosacea	31	MR Egger	1.240	0.111–13.812	0.862		29(0.629)	
			Weighted median	2.143	0.433–10.595	0.350			
			Inverse variance weighted	1.489	0.503–4.400	0.472	0.472	30(0.677)	0.869
			Simple mode	2.448	0.143–41.784	0.541			
			Weighted mode	2.139	0.268–17.070	0.479			
Smoking status: Current	Rosacea	15	MR Egger	6.67E‐11	1.20E‐24–3.70E+3	0.170		13(0.271)	
			Weighted median	0.008	1.12E‐5–6.818	0.163			
			Inverse variance weighted	0.093	4.26E‐4–20.498	0.388	0.472	14(0.220)	0.208
			Simple mode	3.00E‐04	2.54E‐09–44.481	0.205			
			Weighted mode	3.00E‐04	3.43E‐09–32.942	0.194			
Smoking status: Previous	Rosacea	19	MR Egger	1.46E+03	3.99E‐05–5.38E+10	0.423		17 (0.095)	
			Weighted median	64.068	1.385–2.96E+3	**0.033**			
			Inverse variance weighted	84.398	4.040–1.76E+3	**0.004**	**0.016**	18 (0.121)	0.748
			Simple mode	83.954	0.078–8.94E+4	0.228			
			Weighted mode	29.885	0.056–1.58E+4	0.302			

Abbreviation: SNP, single‐nucleotide polymorphism.

The article "Correlation between cigarette smoking and alcohol consumption and Rosacea: A two‐sample Mendelian randomization study" was retracted in 2025. Reasons: compromised peer review; unreliable results or conclusions; concerns about the methods.

**FIGURE 1:** Summary view of the MR images derived from the IVW, MR‒Egger, simple, weighted median and weighted methods. (A) MR results for Cigarettes smoked per day and Rosacea. (B) MR results for Alcoholic drinks per week and Rosacea. (C) MR results for Smoking status: Current and Rosacea. (D) MR results for Smoking status: Previous and Rosacea.

## 4 DISCUSSION

To the best of our knowledge, this is the first MR study on cigarette smoking and alcohol consumption and Rosacea. IVW is the main research method in MR research, and the significance of IVW results indicates that there is a certain significant correlation between them. The results of this study suggest that the number of cigarettes smoked per day and cigarette smoking cessation are associated with Rosacea. The number of cigarettes smoked per day is negatively correlated with the incidence of Rosacea, and cigarette smoking cessation may increase the prevalence of Rosacea. No association was found between alcohol consumption and Rosacea. Meanwhile, sensitivity analysis and horizontal pleiotropy verified the robustness of the main results.

The association of cigarette smoking with alcohol consumption and Rosacea is still controversial. In studies related to cigarette smoking, Suyun Li et al. found that the risk of Rosacea increased in former smokers, while the risk of Rosacea decreased in current smokers.^37^ A case‐control study from the United Kingdom also found that cigarette smoking cessation increased the risk of Rosacea (OR = 1.14, 95%CI: 1.10–1.18).^38^ Y‐X Dai et al. found that cigarette smoking more than 15 cigarettes per day can reduce the probability of Rosacea (OR = 0.51, 95%CI: 0.26–0.99), but his results did not suggest the correlation between cigarette smoking cessation and Rosacea.^16^ In the latest meta‐analysis, it was also believed that cigarette smoking cessation would increase the risk of Rosacea, but the correlation between the number of cigarettes smoked and Rosacea was not analyzed.^39^ On the contrary, Asli Kucukunal et al.’s study suggested that the risk of Rosacea was significantly increased among smokers.^40^ In studies related to alcohol consumption, the latest Meta‐analysis did not find that alcohol consumption was a related risk factor for Rotaria, which was consistent with the results of our study.^10^ However, some cohort studies have found that alcohol intake in women is closely related to Rosacea.^18^ Our findings largely align with those of numerous studies, indicating a notable correlation between cigarette smoking and the onset of Rosacea, while suggesting that alcohol consumption may not be linked to Rosacea. In comparison to other clinical investigations, our results additionally indicate a potential significant association between the quantity of cigarettes smoked daily and the cessation of cigarette smoking with Rosacea, which may help to clarify the risk factors of Rosacea and further understand the occurrence and development of Rosacea. We believe that the number of cigarettes smoked per day reflects the intensity and frequency of cigarette smoking, and current cigarette smoking status reflects whether a person smokes or not. Our results suggested that the number of cigarettes smoked per day increased the risk of Rosacea, while current cigarette smoking status was not associated with Rosacea. This may suggest that the intensity and frequency of cigarette smoking in a population may be a more important indicator of Rosacea prevention than the presence or absence of cigarette smoking.

The article "Correlation between cigarette smoking and alcohol consumption and Rosacea: A two‐sample Mendelian randomization study" was retracted in 2025. Reasons: compromised peer review; unreliable results or conclusions; concerns about the methods.

The mechanism of the correlation between cigarette smoking and rosacea is still unclear, and the vasoconstriction caused by cigarette smoking may be one of the main mechanisms to reduce the incidence of rosacea.^41^ Rosacea as a chronic inflammatory disease.^42^ Nicotine can be used as a treatment for some inflammatory diseases.^43^, ^44^ The anti‐inflammatory and pro‐inflammatory effects of nicotine also play a dual role in inflammatory diseases.^45^ However, lipid oxidation on the skin surface caused by cigarette smoke may change the skin barrier,^46^ further lead to the degradation of collagen, elastic fibers and proteoglycans,^47^ and accelerate the skin aging process.^48^ This could be a possible mechanism for the increased risk of Rosacea after cigarette smoking cessation. There may be some interaction between alcohol consumption and Rosacea, but our results suggest that there is no significant association between alcohol consumption and Rosacea. Further studies are needed to clarify the mechanisms underlying the association between cigarette smoking and drinking and Rosacea.

So far, no study has analyzed the association between cigarette smoking and alcohol consumption and Rosacea using MR. The advantage of our study is that we use large‐scale GWAS data sets for MR analysis. Previous clinical studies have grappled with the challenge of confounding factors influencing research outcomes, potentially undermining the reliability of their findings. To mitigate this issue to some extent, we employed the MR method, which helps attenuate the impact of confounding variables in clinical research. Additionally, we utilized the FDR method to adjust the *P*‐value, thus lowering the likelihood of false positive results. These methodological approaches enhance our confidence in the robustness and reliability of the study outcomes. However, there are some limitations in MR analysis. First, as a data simulation analysis, although we did not find that horizontal pleiotropy occurred, we cannot completely rule out the possibility that horizontal pleiotropy affected our results. Second, because the dataset comes from a public database, we lack a stratified analysis of the data and cannot distinguish factors such as age and sex. Finally, our analysis did not further evaluate the association between cigarette smoking and alcohol consumption and subtypes of Rosacea, which requires further detailed analysis in future work. Our results have some inconsistencies, which may indicate that there is a nonlinear relationship between cigarette smoking and Rosacea. The MR analysis method may not be able to accurately analyze the nonlinear results between the two, and more controlled clinical studies are needed to explore the association between cigarette smoking and Rosacea.

The article "Correlation between cigarette smoking and alcohol consumption and Rosacea: A two‐sample Mendelian randomization study" was retracted in 2025. Reasons: compromised peer review; unreliable results or conclusions; concerns about the methods.

In conclusion, this two‐sample MR analysis found that the number of cigarettes smoked per day and cigarette smoking cessation were associated with Rosacea. The number of cigarettes smoked per day is negatively correlated with the incidence of Rosacea, and cigarette smoking cessation may increase the prevalence of Rosacea. No association was found between alcohol consumption and Rosacea. As a common chronic inflammatory disease in clinical work, Rosacea has a certain impact on the quality of life, self‐esteem and happiness of patients because its clinical symptoms are manifested on the face.^49^ The results of this study are of great help to inform patients with Rosacea to adjust their living habits in clinical work. It also has a guiding role in the prevention and treatment of Rosacea. This study also guides our future exploration of its mechanism.

## CONFLICT OF INTEREST STATEMENT

The author declares no conflicts of interest.

## ETHICS STATEMENT

Not applicable.

## Supporting information

Supporting Information

Supporting Information

Supporting Information

## Data Availability

All the data can be obtained from the open source platform provided in the article. (https://gwas.mrcieu.ac.uk/).
